The article "DNMT3A Regulates miR-149 DNA Methylation to Activate NOTCH1/Hedgehog Pathway to Promote the Development of Junctional Osteosarcoma" was retracted in 2023. Reasons: unreliable results or conclusions; lack of ethics approval or compliance; concerns about the data; concerns about the peer review.

# DNMT3A Regulates miR-149 DNA Methylation to Activate NOTCH1/Hedgehog Pathway to Promote the Development of Junctional Osteosarcoma

**DOI:** 10.1155/2022/3261213

**Published:** 2022-07-21

**Authors:** Shigao Cheng, Wanchun Wang

**Affiliations:** ^1^Department of Orthopedics, Loudi Central Hospital of Hunan Province, Loudi, Hunan, 417000, China; ^2^Department of Orthopedics, The Second Xiangya Hospital of Central South University, Changsha, Hunan, 410011, China

## Abstract

**Purpose:**

To investigate the DNMT3A/miR-149/NOTCH1/Hedgehog axis regulating the development of osteosarcoma.

**Methods:**

First, microRNA and mRNA expression microarrays were downloaded from the GEO database for osteosarcoma and differentially expressed microRNAs were analyzed. Subsequently, we collected cancerous tissues and corresponding paracancerous tissues from 42 osteosarcoma patients and examined the expression levels of miR-149, DNMT3A, and NOTCH1 in the samples. Subsequently, miR-149 was overexpressed in osteosarcoma cells to detect cell proliferation and metastatic ability changes. We then queried the methylation level of the miR-149 promoter on the bioinformatics website and verified it by experiment. We further demonstrated the expression level of miR-149 with NOTCH1 using a dual luciferase assay and confirmed the role of NOTCH1 on osteosarcoma cell growth and metastasis by functional rescue assay. Finally, we detected the activation level of the Hedgehog/catenin signaling pathway by WB and immunofluorescence.

**Results:**

miR-149 was significantly low expressed in osteosarcoma tissues and cells, while DNMT3A and NOTCH1 were highly expressed in osteosarcoma tissues and cells, and negatively correlated with miR-149 expression levels. Overexpression of miR-149 significantly inhibited the growth and metastasis of osteosarcoma cells in vitro and in vivo, and we found that DNMT3A could promote the methylation modification of the miR-149 promoter, thereby inhibiting the expression of miR-149. Subsequently, the experimental results showed that miR-149 could target negative regulation of NOTCH1, and further overexpression of NOTCH1 in cells with high miR-149 expression could promote the growth and metastasis of osteosarcoma cells in vitro.

**Conclusion:**

The methyltransferase DNMT3A suppresses miR-149 expression by promoting methylation modification of the miR-149 promoter, resulting in elevated expression levels of NOTCH1 in cells, therefore exacerbating activation of the Hedgehog signaling pathway and therefore exacerbating the development and progression of osteosarcoma.

## 1. Introduction

Osteosarcoma (OS) is the most frequent malignant bone tumor in children and adolescents, and it mostly affects the metaphysis of long bones [1]. The annual incidence of OS varies between 1 and 4 per million, with men having a slightly greater prevalence than women [2]. Despite the low overall prevalence of OS, the prognosis is dismal. The 5-year survival rate for patients without metastases is approximately 65–70 percent when limb salvage surgery and neoadjuvant chemotherapy are combined [3]. Because osteosarcoma has such a dismal prognosis following metastasis, new therapeutic approaches are desperately needed [4].

Long noncoding RNAs (lncRNAs) with more than 200 nucleotides are thought to regulate protein-coding genes in various ways, including epigenetic regulation, transcription regulation, posttranscriptional regulation, and microRNA (miRNA) regulation [5–7]. MicroRNAs (miRNAs) are single-stranded RNAs with a length of 21-25 nucleotides that do not code for proteins. Its expression alterations are linked to the tumor's occurrence, progression, diagnosis, and prognosis [8]. It is worth noting that miRNAs have a unique property: they are extremely stable in plasma and serum and are not destroyed by RNase [9]. Finding miRNA biomarkers with unique expression patterns will be critical for the early detection and treatment of OS.

It has been demonstrated that odd DNA methylation regulates carcinogenesis and the course of many cancers. According to growing data, tumorigenesis is linked to strange epigenetic variables such as DNA methylation, histone modification, RNA m6A modification, RNA binding proteins, and transcription factors. [10] Methylation of RNA, notably m6A modifications of RNA, and histone modifications, which are thought to be the essential contributors to cancer development, are among the critical epigenetic alterations in cancer development [11]. DNMT3A (NM 022552.4) belongs to the DNA methyltransferases (DNMTs) family, which catalyzes the addition of a methyl group to the 5-cytosine residue CpG dinucleotides. The DNMT3A gene (2p23.3) encodes a protein that methylates previously unmethylated genomic DNA and is responsible for genome-wide de novo DNA methylation [12]. DNMT3A also acts as a transcriptional corepressor, suppressing gene transcription without the need for its de novo methyltransferase activity [13, 14]. It is frequently mutated in AML and has been linked to a poor prognosis; however, DNMT3A mutations in solid human tumors have not been well studied [15]. Although DNA methylation patterns in OS have attracted attention as an essential biomarker and therapeutic target, the mechanism of regulation of OS by DNMT3A with miR-149 and DNA methylation remains unclear. miR-149 is further overexpressed in cells with NOTCH1, and the growth and metastasis of the resulting tumor cells are also unclear, so tumor recurrence and widespread metastasis also complicates the clinical treatment of osteosarcoma. To date, the molecular mechanisms underlying the malignant biological behavior of osteosarcoma remain unclear, although molecular biology studies associated with osteosarcoma have provided a theoretical basis for its pathogenesis. Exploring the pathogenesis of OS is important for improving diagnosis and finding new therapeutic targets. Therefore, in our study, a functional enrichment study was carried out to investigate the possible mechanisms.

## 2. Materials and Methods

### 2.1. Bioinformatics Analysis

The Gene Expression Omnibus (https://www.ncbi.nlm.nih.gov/geo/) was used to download osteosarcoma-related gene expression datasets (DEGs). Three gene expression datasets were obtained: one miRNA (GSE67268) and two gene expression datasets (GSE29001 and GSE20347). Normalized expression data were used to screen DEGs and differentially expressed miRNAs using the limma package (http://master. http://bioconductor.org/packages/release/bioc/html/limma.html) with |log2FC| > 1.5 and adj.*P*.Val = 0.05. Also, pheatmap (https://cran.r-project.org/web/packages/pheatmap/index.html) was used to create a miRNA heat map. The target genes of differentially expressed miRNAs were predicted using the starBase, TargetScan, and mirRDB databases. jvenn (http://jvenn.toulouse.inra.fr/app/example.html) was also used to screen differentially expressed miRNAs (GSE29001 and GSE20347). The HPA website was utilized to retrieve the staining intensity of DNMT3A and NOTCH1 for immunohistochemistry in normal esophageal tissue and osteosarcoma tissue samples.

### 2.2. EdU Staining

Osteosarcoma cells in the logarithmic growth phase were seeded in triplicate into 96-well plates at 4 104 cells/well. After 24 hours, the cells were treated with various chemicals. 2 hours in EdU media at 100 l/well, followed by 100 l/well cell fixative, 2 mg/ml glycine, and 100 l/well permeabilizer (phosphate-buffered saline (PBS) containing 0.5 percent Triton X-100). Incubation with antifluorescence quenching blocking solution (100 l/well) followed by staining with Apollo and Ho osteosarcoma hst 33342 reaction solutions. The number of EdU-stained cells was counted using microscope images. Positive cells have red nuclei. In order to obtain the EdU staining rate (%), the number of positive cells was divided by (number of positive cells + number of negative cells) 100 percent.

### 2.3. Colony Formation

Cells were cultured at a density of 1 × 10^3^ cells/well in 90 mm cell culture dishes containing 5 ml of complete DMEM complete +10% FBS. All culture dishes were incubated in a sterile incubator at 37°C and 5% CO_2_ for 2 weeks. The culture medium was changed every two days. Cells were washed three times with PBS to remove residual cells and then fixed with 4% formaldehyde for 10 min at room temperature. The cells were then stained with crystal violet (0.1%) for 10 minutes at room temperature. The colonies were counted under a light microscope. A population of >50 cells was considered a clone.

### 2.4. Caspase-3 Activity Assay

MG63 or TE-3 cells were transfected in 100 l of media in 96-well flat-bottomed microplates. Then, 100 l Caspase-Glo 3/7 Reagent (Promega, Madison, WI, USA) was added to each well and shaken for 1-2 minutes, 3 h incubation at ambient temperature. A microplate reader measured 485Ex/527Em fluorescence (PerkinElmer, Waltham, MA, USA). The apoptotic index is the ratio of apoptotic nuclei to total cells in each group.

### 2.5. Apoptosis Test

Apoptosis was detected using the Annexin V-FITC/Propidium Iodide Apoptosis Detection Kit (BD Biosciences, San Diego, CA, USA). MG63 and SAOS-2 cells were plated in 6-well plates at 3105 cells per well, collected, washed twice with PBS, resuspended in binding buffer, and stained with Annexin V-FITC and PI. Staining cells for 15 minutes at 4°C in the dark, then analyzing using a B osteosarcoma kman Coulter flow cytometer (B osteosarcoma kman Gallios, Fullerton, CA, USA).

Transwell MG63 and SAOS-2 cells were collected and resuspended in 1 105 cells/ml serum-free DMEM. 200 l of sample was introduced to 8 m Transwell chambers precoated with Matrigel. The Transwell chambers were then placed in a 24-well plate with 500 l DMEM (10% FBS) in each well. Affixated cell membranes from Transwell chambers were collected. Upper surface cells were gently scraped off with a cotton swab, while lower surface cells were gently washed with PBS. After fixing with 4 percent paraformaldehyde, the cells were stained with 0.1 percent crystal violet for 20 minutes at room temperature. The invading cells were counted under a light microscope (Olympus, 200x).

### 2.6. Tumorigenesis In Vivo

Our Animal Care and Use Committee approved all animal experiments. We injected miR-149 mimic or control transfected MG63 or SAOS-2 cells (7106) into 4-week-old nude mice. Every 5 days, the tumor volume was measured 5 times. Then, the mice were killed and the tumors weighed. Tumor samples were also preserved at -80°C for histological analysis.

### 2.7. Immunohistochemistry

Xenograft tumors were collected and sectioned. In order to quench endogenous peroxidase, the 4 m thick sections were deparaffinized, rehydrated, and then labeled with antibody overnight at 4°C, followed by 30 seconds of hematoxylin counterstaining and slipcovering with secondary streptavidin-horeradish peroxidase-conjugated antibody (Santa Cruz Biot Osteosarcoma h, Santa Cruz, CA).

### 2.8. TUNEL Stain

Tumor sections were stained with 4′,6-diamidino-2-phenylindole (DAPI, 1 : 5000; Beyotime, China) and TUNEL kit to evaluate apoptosis-related alterations (Roche, Basel, Switzerland). We also counted TUNEL-positive cells using a laser scanning confocal microscope (SP8, Leica, Japan).

### 2.9. MSP-qPCR

The DNA Methylation Kit (TIANGEN Biot Osteosarcoma h, Beijing, China) was used to modify human genomic DNA with bisulfite (Zymo Research, Orange, CA, USA). The modified DNA (1 g) was amplified using Winkybio (Guangzhou, China) MSP methylation and nonmethylation primers. 45 seconds each at 95°C, 62°C, and 72°C with a final extension of 10 minutes at 72°C. qPCR was used to test PCR products.

### 2.10. Assay for Luciferase

WT NOTCH1-3′ untranslated region (UTR) (PGLO-NOTCH1-WT) and MUT NOTCH1 sequence with MUT miR-149 binding site (PGLO-NOTCH1-MUT) were purchased from Guangzhou Land Bio (Guangdong, China). Positive control was renilla luciferase plasmid pRL-TK. They were cotransfected with miR-149mimic and NC mimetic in HEK-293 T cells at 70-80% confluence. Transfection was performed using the following ratios of firefly luciferase reporter vector: mimic: pRL-TK = 0.50 nM: 0.1 g. Lysed cells were tested utilizing the Dual-Luciferase® Reporter Vector Assay System (E1910, Promega, Madison, WI, USA) The relative luciferase activity was calculated as the ratio of firefly luciferase to ranelia luciferase activity.

### 2.11. Immunofluorescence

Fixed with prechilled acetone, cells on glass coverslips were rerinsed three times with PBS and then reincubated in 10% goat serum with 0.3 percent hydrogen peroxide, followed by overnight incubation with primary antibodies to atenin (both from Abcam). A secondary HRP-conjugated antibody (ZSGB-BIO, Xicheng, Beijing, China) was then incubated for 45 minutes at room temperature. DAPI was used to stain the nuclei (Boster Biot osteosarcoma technology, Wuhan, China).

### 2.12. Data Analysis Methods

SPSS was applied for statistical analysis. The data was noted as “mean ± standard deviation.” Chi-square test or Student *t*-test was applied for two-sample comparisons. All the tests at *P* value < 0.05 were considered a significant difference.

## 3. Experimental Results

### 3.1. miR-149 Is Significantly Underexpressed in Osteosarcoma Tissues and Cells

The GEO database contained 113 osteosarcoma tumor samples and normal esophagus tissues. We analyzed 63 differently expressed microRNAs (normal vs. cancer) (Figure 1(a)), of which miR-149 expression was most significantly downregulated in osteosarcoma tissues. We then looked at miR-149 expression in 42 osteosarcoma patients' tumors and paraneoplastic organs. Tumor tissues had significantly reduced expression of miR-149 (Figure 1(b)), and we investigated the connection between miR-149 expression and clinical stage, lymph node metastasis, and differentiation levels of osteosarcoma patients. The expression of miR-149 was found to be significantly lower in Stage III and IV patients than in Stage I and II patients (Figure 1(c)), and in lymph node metastasis patients than in nonmetastasis patients (Figures 1(d) and 1(e)). qRT-PCR evaluated miR-149 expression in normal human esophageal epithelial cells HET-1A and osteosarcoma cell lines SAOS-2, 9706, and MG63 (Figure 1(f)). So, we wondered if decreased miR-149 expression was linked to osteosarcoma formation and progression.

### 3.2. Exogenous Overexpression of miR-149 Significantly Inhibits the Growth and Metastasis of Osteosarcoma Cells In Vitro

We transfected miR-149 mimic into MG63 and SAOS-2 cells to confirm the effect of miR-149 on osteosarcoma cell proliferation and development (Figure 2(a)). After transfection with miR-149, the number of cell clones generated by MG63 and SAOS-2 cells was dramatically reduced (Figure 2(b)). Using a caspase-3 kit and flow cytometry, we discovered that miR-149 mimic dramatically increased caspase-3 activity in KYSE-15O and SAOS-2 cells (Figures 2(c) and 2(d)). Using qRT-PCR, we discovered that miR-149 raised E-cadherin and ZO-1 mRNA expression levels while decreasing N-cadherin and vimentin mRNA expression levels (Figure 2(e)), indicating that miR-149 promotes EMT. Using the Transwell experiment, we confirmed our suspicions: miR-149 transfection reduced the migratory and invasion abilities of MG63 and SAOS-2 cells (Figures 2(f) and 2(g)). In vitro, miR-149 appears to slow osteosarcoma cell growth and metastasis.

### 3.3. The miR-149 Promoter Has Significant Methylation Modifications

To clarify the upstream regulatory mechanism of miR-149, we first found that miR-149 belongs to a transcript with HYC gene (Figure 3(a)), and we found that the promoter sequence of miR-149 has a distinct CpG island (Figure 3(b)). Thus, we speculated whether it was because the miR-149 promoter was modified by methylation in osteosarcoma, thus suppressing its expression. To test our conjecture, we harvested the methylation level of miR-149 promoter in 42 osteosarcoma patients by MSP-qPCR. We found that the methylation level of miR-149 promoter was significantly higher in cancer tissues than in paracancerous tissues (Figure 3(c)). Moreover, we further analyzed that the expression level of miR-149 was negatively correlated with its methylation level in 42 osteosarcoma tumor samples (Figure 3(d)). And we also found that the methylation modification level of miR-149 promoter was significantly lower in normal human esophageal epithelial cells HET-1A than in osteosarcoma cell lines (Figure 3(e)). Moreover, we further found that the expression level of miR-149 in the cells was significantly increased after treatment with 5-aZa-CDR on the osteosarcoma cell line (Figure 3(f)).

### 3.4. DNMT3A Promotes Methylation Modification of miR-149 Promoter

We found in result 4 that the miR-149 promoter has significant methylation modifications, thereby repressing its transcription, which leads to the growth and metastasis of osteosarcoma cells. To determine which specific methyltransferase initiates the role, we focused on DNMT1, DNMT3A, DNMT3A, and DNMT3L. We first examined the expression levels of these four genes in 42 paired osteosarcoma tissues and paracancerous tissues and found that they all had significantly high expression in osteosarcoma tissues (Figure 4(a)), and we further found that the expression levels of DNMT1, DNMT3A, DNMT3B, and DNMT3L were higher in cancer tissues than in normal esophageal tissues, but there was no significant difference, while the expression level of DNMT3A was significantly higher in osteosarcoma tissues than in normal esophageal tissues (Figure 4(b)). Therefore, we further analyzed the correlation between miR-149 and DNMT3A in 42 osteosarcoma patients, and we found that miR-149 had a significant negative correlation with DNMT3A (Figure 4(c)). We further found in the HPA site that DNMT3A staining intensity was significantly higher in osteosarcoma tissues than in normal esophageal tissues (Figure 4(d)). To further determine that DNMT3A promotes the methylation modification of miR-149, we first examined the binding relationship between DNMT3A and miR-149 promoter in osteosarcoma cell lines by ChIP-qPCR assay, and we found that the enrichment level of miR-149 promoter in the complexes pulled down using anti-DNMT3A antibody was significantly higher than that of IgG (Figure 4(e)). Moreover, we further constructed a luciferase reporter vector pGL3-enhancer containing miR-149 promoter and cotransfected it with different doses of DNMT3A overexpression plasmids into 293T cells, and we found that the luciferase activity in 293T cells decreased significantly with the increase of DNMT3A overexpression plasmid dose (Figure 4(f)). The above results suggest that DNMT3A can bind to miR-149 promoter to promote its methylation modification, thus inhibiting the expression of miR-149.

## 4. Discussion

OS is the most prevalent malignant bone tumor, and it has a significant impact on patients' quality of life and life expectancy. Early detection and treatment of osteosarcoma patients cannot be overstated [16]. It has an early onset age, a high malignancy, a high rate of metastasis, and a bad prognosis [17]. Its proclivity for metastasizing is the most common cause of therapy failure and poor prognosis [18]. Despite significant advances in surgery and neoadjuvant treatment, most patients still have a dismal prognosis. Some researchers have attempted to apply gene treatments to OS in recent years, including adenovirus-based gene transfection and siRNA-based gene silencing [19–21], and it is now making progress in certain basic studies. Since the discovery of miRNA, researchers from all around the world have been exploring its involvement in malignancies. Some miRNAs have been discovered to promote or repress malignancy in tumors [22, 23].

lncRNAs are primarily found in the cytoplasm, acting as a miRNA sponge [24]. For patients with osteosarcoma, there are currently few biomarkers with high sensitivity. Bioinformatics research in the past was frequently limited to a single database or single gene prognostic value, which has limits. In recent decades, scientists have uncovered many factors of epigenetic modification influencing gene expression that interfere with tumor formation [25, 26]. DEGs are primarily engaged in DNA replication, mitosis, and cell cycle regulatory signaling pathways, according to the GSEA data. DNA replication is the cellular activity that most easily leads to cancer, and genome instability is a marker of cancer [27].

Abnormal mitosis can promote the unrestricted expansion of faulty cells, making it the most common way for tumors to form [28]. Cell cycle dysregulation is the cause of aberrant cell proliferation, which is a hallmark of cancer, and the loss of cell cycle checkpoint control promotes genetic instability [29].

In our study, firstly, we analyzed the expression levels of miR-149 in the tumor tissues and corresponding paracancerous tissues of 42 patients with osteosarcoma and confirmed that miR-149 was significantly low expressed in osteosarcoma tissues and cells; secondly, to further verify the effect of miR-149 on the growth and development of osteosarcoma cells, the expression levels of EMT-related proteins in the cells were detected by qRT-PCR, and we found that exogenous overexpression of miR-149 significantly inhibited the growth and metastasis of osteosarcoma cells in vitro. Next, our experiments confirmed that miR-149 can significantly inhibit the growth of osteosarcoma cells in vivo and that the upstream of miR-149 has a regulatory mechanism, which suggests that the miR-149 promoter has significant methylation modifications. Then, miR-149 promoter represses its transcription, leading to osteosarcoma cells' growth and metastasis. We focused on DNMT1, DNMT3A, DNMT3A, and DNMT3L, and we found that DNMT3A promotes miR-149 promoter methylation modification. Finally, to clarify the downstream regulatory mechanisms of miR-149, we confirmed that miR-149 targets the negative regulation of NOTCH1 expression and NOTCH1 promotes osteosarcoma cell progression through activation of the Hedgehog signaling pathway, thus exacerbating the development and progression of osteosarcoma.

Consistently, in OS tissue and cells, the DNA methyltransferase inhibitor 5-AZA-dC decreased DNA methylation in the APCDD1 promoter and restored APCDD1 expression. Furthermore, DNMT3a was the primary DNA methyltransferase that promoted hypermethylation of DNA in the APCDD1 promoter, lowering APCDD1 mRNA levels in OS tissues, but not DNMT1 or DNMT3b [30]. Thus, the present study shows that we provide for the first time that miR-149 is significantly low expressed in osteosarcoma tissues and cells, while DNMT3A and NOTCH1 are highly expressed in osteosarcoma tissues and cells. Thus exacerbating the development and progression of osteosarcoma. DNMT3A is involved in important cancer-related biological processes in OS.

### 4.1. Limitation

This is a study to develop predictive features for osteosarcoma based on epigenetically modified genes. However, our study has some limitations [31]. First, further confirmation of the efficacy of this study in additional independent prospective trials with functional testing of the identified genes is needed in this study. In addition to this, we need more prospective clinical studies and larger sample sizes to evaluate the diagnostic performance of this prognostic model. Therefore, more work remains to be done before the results can be applied to clinical practice.

## 5. Conclusion

Our study created a novel epigenetically relevant gene signature that has demonstrated significant clinical utility in predicting OS in patients with osteosarcoma. The methyltransferase DNMT3A exacerbates osteosarcoma development and progression by promoting methylation modification of the miR-149 promoter, thereby repressing miR-149 expression and leading to elevated levels of NOTCH1 expression in cells, thereby promoting activation of the Hedgehog signaling pathway. This signature may serve as a reliable biomarker for early detection and prognosis of osteosarcoma.

## Figures and Tables

**Figure 1:** miR-149 was significantly low expressed in osteosarcoma tissues and cells. (a) Differentially expressed microRNA in microRNA expression microarray GSE67268 of osteosarcoma tissues. (b) qRT-PCR detection of miR-149 expression levels in cancer tissues and paired paraneoplastic tissues of 42 osteosarcoma patients. (c–e) Analysis of miR-149 451a expression levels in relation to clinical stage, lymph node metastasis, and differentiation level of osteosarcoma patients. (f) miR-149 expression levels in normal human esophageal epithelial cells HET-1A and osteosarcoma cell lines SAOS-2, osteosarcoma 9706, and MG63. In (b–e), each point represents one sample, and data were analyzed for differences using the paired or unpaired test; ^∗∗^*P* < 0.01, ^∗∗∗^*P* < 0.001. In (f), data were analyzed for differences using one-way ANOVA and Tukey's multiple comparison test for analysis of variance on data; ^∗∗∗^*P* < 0.001.

**Figure 2:** Exogenous overexpression of miR-149 significantly inhibits the growth and metastasis of osteosarcoma cells in vitro. (a) qRT-PCR to detect the expression level of miR-149 in MG63 and SAOS-2 cells after transfection with mimic control or miR-149 mimic. (b) Plate cloning assay to detect the number of clones formed in MG63 and SAOS-2 cells. The number of clones formed. (c) Caspase-3 kit to detect changes in caspase-3 activity in MG63 and SAOS-2 cells. (d) Flow cytometry to detect the proportion of apoptosis in MG63 and SAOS-2 cells. (e) qRT-PCR to detect the EMT-related factors E-cadherin, ZO-1, vimentin, and N-cadherin mRNA expression levels. (f, g) Transwell assay to detect the migration and invasion ability of MG63 and SAOS-2 cells. Each experiment was repeated three times, and data were presented as mean plus or minus standard deviation, and in (a–g), 2-way ANOVA and Tukey's multiple comparison test were used to analyze the data for differences, ^∗∗∗^*P* < 0.001.

**Figure 3:** miR-149 promoter has significant methylation modification. (a) MSP-qPCR detects the methylation level of miR-149 promoter in cancerous and paraneoplastic tissues of 42 osteosarcoma patients. (b) Correlation between miR-149 and its DNA methylation level in tumor tissues of osteosarcoma patients. (c) MSP-qPCR detects the correlation between miR-149 and its DNA methylation level in normal tissues of osteosarcoma patients. Methylation levels of the promoter of miR-149 in tumor tissues from osteosarcoma patients. (d) Correlation between miR-149 and its DNA methylation levels in tumor tissues from osteosarcoma patients. Each point in CD represents one sample, and the data were tested for significant differences using the paired *t*-test, ^∗∗^*P* < 0.01. In (e, f), each experiment was repeated three times, and the data were presented as mean plus or minus standard deviation, using one-way or 2-way ANOVA and Tukey's multiple comparison test for analysis of variance on data, ^∗∗^*P* < 0.01, ^∗∗∗^*P* < 0.001.

**Figure 4:** DNMT3A promotes miR-149 DNA methylation modification. (a) Pearson correlation test to analyze the correlation analysis between miR-149 and DNMT3A expression levels. (b) HPA website to retrieve the staining intensity of DNMT3A in normal esophageal tissues and osteosarcoma tissue samples by immunohistochemistry. (c) ChIP-qPCR to detect DNMT3A binding relationship with miR-149 promoter. (d) The luciferase reporter vector pGL3-enhancer containing miR-149 promoter was constructed, cotransfected into 293T cells with different doses of DNMT3A overexpression plasmids, and the expression level of miR-149 in the cells was detected. In (a), each point represents one sample, and the data were tested for significant differences using paired *t*-test, ^∗∗^*P* < 0.01. In (e, f), each experiment was repeated three times, and the data were presented as mean plus minus standard deviation using one-way or 2-way ANOVA and Tukey's multiple comparison test for analysis of variance on data; ^∗∗^*P* < 0.01, ^∗∗∗^*P* < 0.001.

## Data Availability

All data generated or analyzed during this study are included in this published article.
